The article "A scientometric analysis approach on the plastic sand" was published in 2023. Journal: Heliyon.

# A scientometric analysis approach on the plastic sand

**DOI:** 10.1016/j.heliyon.2023.e14457

**Published:** 2023-03-11

**Authors:** Bawar Iftikhar, Sophia C. Alih, Mohammadreza Vafaei, Raid Alrowais, Muhammad Tariq Bashir, Alamgir Khalil, Muhammad Rizwan, Muhammad Faisal Javed, Muhammad Faisal Rehman, Abdullah Mohamed

**Affiliations:** a School of Civil Engineering, Universiti Teknologi Malaysia, 81310 Johor Bahru, Johor, Malaysia; b Institute of Noise and Vibration, School of Civil Engineering, Universiti Teknologi Malaysia, 81310 Johor Bahru, Johor, Malaysia; c Department of Civil Engineering, Jouf University, Al-Jawf 72388, Saudi Arabia; d Department of Civil Engineering, CECOS University of IT and Emerging Sciences, Peshawar 25000, Pakistan; e Department of Civil Engineering, University of Engineering and Technology, Peshawar 25120, Pakistan; f National Institute of Transportation Risalpur National University of Sciences & Technology, Islamabad, Pakistan; g Department of Civil Engineering, COMSATS University Islamabad, Abbottabad Campus, 22060, Pakistan; h Department of Architecture, University of Engineering and Technology Peshawar, Abbottabad Campus, Pakistan; i Research Centre, Future University in Egypt, New Cairo 11835, Egypt

**Keywords:** Waste material, Sustainable material, Scientometric analysis, Waste management, Plastic waste, Sand

## Abstract

The purpose of this research was to conduct a scientometric evaluation of the literature pertaining to plastic sand in order to evaluate its many aspects. Conventional review studies have several limitations when it comes to their capacity to completely and properly link different sections of the published research. Some of the more complicated features of advanced research are co-occurrence analysis, science mapping and co-citation analysis. During the study, the most inventive authors/researchers renowned for citations, the sources with the largest number of publications, the actively involved domains, and co-occurrences of keywords in the research on plastic sand are investigated. This study is limited to scientometric analysis of the available literature data on plastic sand. The VOSviewer application (version 1.6.18) was used to perform the analysis after bibliometric data for 4512 publications were extracted from the Scopus database and utilised in the extraction process from the year 2021 to June 2022. With the support of a statistical and graphical description of researchers and nations that are contributing, this study will aid researchers in the establishment of collaborative ventures and the exchange of fresh techniques and ideas with one another.

## 1 Introduction

Plastic waste, such as plastic bottles, bags, and sheets, cannot be easily biodegraded, making it one of the most difficult kinds of pollutants to eliminate. Global plastic waste annually reaches 25 million tonnes [1]. According to the United Nations Development Program, only around 10% of plastic garbage was recycled between 1950 and 2015; the remainder was thrown away in landfills or somewhere else in the environment (2019). Fig. 1 depicts the development of plastic garbage from 1950 to 2019 [2]. The existing consumption patterns and methods of waste management will result in around 12,000 million tonnes of litter made of plastic being dumped in landfills and the natural environment by the year 2050, making it one of the most difficult kinds of pollution to eliminate [3]. Thus, there have been several initiatives worldwide, particularly in industrialised nations, to transform plastic trash into valuable items [4]. Since the construction sector dominates the majority of countries and consumes the most raw resources [5], there is enormous opportunity for generating new building components from the waste plastic.

The article "A scientometric analysis approach on the plastic sand" was published in 2023. Journal: Heliyon.

**Fig. 1:** Generation of global plastic waste from 1950 to 2019 [3].

The replacement of commonly used construction materials such as concrete (cement) blocks and plastic sand bricks or blocks might help to a reduction in cement use and the accompanying CO_2_ pollution. The cement industry's contribution to the atmosphere in the form of carbon dioxide emissions is amongst the greatest of all industries [6], with cement production accounting for 8–10% of worldwide CO_2_ emissions [7].

The level of demand for sand was three times higher 20 years ago than it is today [8]. The rate of rise in requirement for sand has been tremendous, exceeding 18 kg of sand per individual per day. Sand and gravel are estimated to account for 43% of the world's total material extraction in 2009 [9], with 87% of that amount being taken from terrestrial sources including quarries and pits [10]. Using remote sensing techniques, researchers calculated that extraction rates at Lake Poyang in China reached 488 Mt over the period of 2005–2006 [11]. Lake Poyang is the largest known region of sand mining operations anywhere in the world. Increasing levels of income and consumption, as well as a quickening pace of commerce, are the primary factors behind this rise [12]. The demand for sand in construction and infrastructure has increased at a rate of 4.5% annually over the past decade, and this sector is currently responsible for 75% of all sand consumption [13]. Since 1990, the consumption of sand in the emerging regions of the Asia-Pacific area has enhanced at an average yearly growth rate of 6.5% [13], while consumption has levelled out in Europe and North America. Sand utilisation is predicted to grow at 30.8 times larger in the year 2090 comparing to the decade of 2020 [14] if significant attempts are undertaken to achieve carbon neutrality by the year 2100. This is because investment in massive development such as hydropower facilities demands large amounts of sand [15].

The article "A scientometric analysis approach on the plastic sand" was published in 2023. Journal: Heliyon.

The global demand for sand has grown, in part as a result of population growth, rising living standards, and fast urbanization [16,17]. Sand is utilised in a variety of businesses and goods [18], including as water filtration, polymers, and the electronics industry [16]. Practically each structure, dam, road, wine glass, and mobile phone has sand-related substance [19]. For the purpose of extracting oil from shale, the fracking sector makes use of enormous quantities of frack sand. Consequently, the United Nations Environment Programme (UNEP) has considered sand to be one of the natural resources that has the highest reported level of use at the present time [19]. According to a UNEP analysis, sand and gravel accounted 85% of the weight of minerals produced annually [20]. The widespread utilisation of sand is unsustainable, posing an additional environmental concern [21]. According to the UNEP (2019), one of the greatest obstacles to sustainability in the 21st is the exploitation of sand and gravel. In many places, however, these materials are one of the least supervised of all harvested and marketed resources. Thus, rivers, river deltas, and shoreline deteriorate, while sand mafias make a profit and its supply rises [22]. Plastic sand is an ecofriendly material due to the ease with which it can be recycled, in contrast to sand cement (concrete), the recycling of which is significantly more challenging and less economically feasible.

Several research and assessments on the usage of the plastic waste in the construction industry have been conducted in recent years, and the findings have been promising [[4], [7], [8], [13], [22], [23], [24], [25], [26], [27], [28], [29], [30], [31], [32], [33], [34], [35], [36], [37], [38], [39], [40]]. In the past, the reuse of waste plastics as construction materials in developing nations has been investigated. The mechanical qualities of polyethylene terephthalate (PET) bottles filled with sand or soil make them appropriate for use in wall and slab construction [41]. Additionally, studies has been done on the use of waste from plastic with sand to generate additional construction material like bricks and blocks, which might be used to reduce plastic pollution [[42], [43], [44], [45]]. Eco-bricks may also be created by filling plastic bottles with plastic food wrappers [46]. As aggregate for lightweight concrete, waste plastics were utilised [47,48]. The use of plastic-coated aggregates in the production of asphalt permits a 10% decrease in bitumen use [49]. Plastic fibres are a cost-effective, corrosion-resistant option for reinforcing concrete [47]. For the soil, to enhance its energy absorption capacity and the compressive strength PET fibres have been utilised [50]. In addition, a number of research [[51], [52], [53], [54], [55], [56]] have focused on the incorporation of plastic waste into industrial sector to enhance its physical properties. In nations such as the USA and the UK, much study has been undertaken on the addition of plastic trash to concrete mix [51,[57], [58], [59], [60]]. Other research have investigated the use of sand-filled plastic bottles as a construction technique [56]. The concept of creating a building material by combining plastics and concrete dates back to the 1980s. The United States Patent and Trademark Office issued a patent involving the combination of plastic and concrete in 1986 [51].

The article "A scientometric analysis approach on the plastic sand" was published in 2023. Journal: Heliyon.

As a result of growing environmental concerns, scientists are doing increasingly in-depth research on plastic sand. However, they are running against informational hurdles that may make it difficult for them to conduct creative research or work together with other academics. As a consequence of this, it is of the utmost importance to devise and put into action a method that provides researchers with the opportunity to get essential evidence from the sources available that is most reliable. A scientometric approach executed with the help of the software programme, might be of assistance in making up for this shortcoming. A scientometric examination of the bibliographic records that have been published on plastic sand up to June 2022 is going to be carried out as part of this research. By utilising the suitable software tool, a scientometric analysis is able to quantitatively evaluate massive amounts of bibliometric data. Conventional review studies are unable to accurately and thoroughly link disparate elements of the published research. Mapping scientific phenomena, identifying co-occurrences, and citing related research are some of the most demanding components of modern research. With the use of scientometric analysis, it is also possible to identify sources with keyword co-occurrence, the principal authors according to articles and citations, the most active research regions, and the most research publications in plastic sand. The VOSviewer application was employed to conduct the analysis after bibliometric data from 4512 relevant articles was extracted from the Scopus database and utilised. This scientometric analysis will help researchers to build alliances and exchange novel concepts and approaches because of the graphical and statistical representation of countries and authors that is included in it.

The article "A scientometric analysis approach on the plastic sand" was published in 2023. Journal: Heliyon.

## 2 Methods

This study performed scientometric analysis [[61], [62], [63]] on the bibliographic data in order to quantitatively evaluate the various characteristics of the bibliographic data. A reliable search engine is essential because so many articles have been written on the subject matter. For this endeavour, Scopus and Web of Science are two highly specialised search engines that are ideal because of their accuracy [64,65]. Scopus, which is strongly advised by researchers [66,67], was utilised to gather bibliographic material for this inverstigation on the plastic sand. As of June 2022, search on Scopus for “plastic sand” yielded 8674 articles. In order to remove any papers that were not essential, many filter settings were utilised. The following kinds of documents were considered for inclusion in the study namely: (a) journal articles, (b) conference papers, (c) journal reviews, and (d) conference reviews. The source types “journal” and “conference proceedings” were selected. The “year of publication” limitation was set from “2000 to 2022” and the “language” restriction was specified to “English” The “subject areas” of “engineering”, “material science”, and “environmental science” were chosen for further research. After applying these conditions, a total of 4512 records were maintained. In a similar fashion, a number of research investigations have been carried out by making use of the same technique [[68], [69], [70]].

Studies in scientometry make use of a methodology known as scientific mapping, which was created by researchers for the purpose of bibliometric data processing [71]. Records from Scopus were saved in a format known as Comma-Separated Values, or CSV files, in order for them to be analysed using the appropriate tools. The scientific visualisation of the material that was gathered and the quantitative analysis of it were both constructed with the help of VOSviewer (version 1.6.18). VOSviewer is a mapping tool that is easily available, based on open source software, and is utilised in a broad variety of disciplines. Academics [[72], [73], [74], [75], [76]] strongly advocate using this programme. Because of this, the goals of this study might be considered accomplished thanks to the application of VOSviewer. The CSV files that were generated were imported into VOSviewer, and additional analysis was carried out while ensuring that the data's integrity and consistency were not compromised. During the bibliographic review, we looked at the publishing sources, the keywords that were used the most often, the academics who had the most publications and citations, and the countries that were involved. The numerous characteristics, as well as their interrelationships and co-occurrence, were depicted visually, and the statistical information on those characteristics was provided in tables. Fig. 2 illustrates the scientometric strategy's flowchart.

The article "A scientometric analysis approach on the plastic sand" was published in 2023. Journal: Heliyon.

**Fig. 2:** Scientometric strategy's flowchart.

## 3 Analysis

### 3.1 Subject areas and annual publications

This research was conducted using the Scopus analyzer to identify the most relevant study fields. As seen in Fig. 3, Engineering on top, Materials Science on second and Environmental Science finally were determined to be the top 3 recorded in this field, with about 32.5%, 17.1%, and 13.9% of documents, accounting for a total 63.5% contribution based on the total number of documents. In addition, as seen in Fig. 4, the Scopus database was analysed to determine the kind of publications containing the searched phrase. This study revealed that (i)-journal articles, (ii)-conference papers, (iii)-journal reviews, and (iv)-conference reviews recorded for around 74.5%, 22.6%, 1.8% and 1.1% of all materials, respectively. Fig. 5 illustrates the yearly publishing trends in the field of subject research from 2001 to 2022. As it can be seen that from 2001 to 2017, there was a steady growth in the number of publications, which averaged around 100 per year. During the last four years (2018–2021), the number of publications climbed dramatically, averaging about 370 per year on average, whereas up to mid of this year 2022 i.e. June 2022, the publication growth has already been reached around 250 and still many more will come by the end of this year by seeing this trend.

**Fig. 3:** Articles by subject areas.

**Fig. 4:** Type of document related to study field.

**Fig. 5:** Annual article publishing trend.

### 3.2 Publication sources

The sources of publishing are found using VOSviewer based on the obtained bibliographic data. “Bibliographic coupling” was choosen as the “type of analysis” and “sources” were maintained as the “unit of analysis” during the study. At a minimum of 15 papers were assigned to each publication source, and 24 of the 563 publication sources satisfied this requirement. Table 1 displays the publishing sites that released at least 15 publications on plastic sand from 2001 to June 2022, including the total number of citations count collected within this time frame. “Construction and building materials”, “marine pollution bulletin”, IOP conference series: materials science and engineering”, “soil dynamics and earthquake engineering” and “IOP conference series: earth and environmental science” contain 134, 63, 56, 53 and 49 papers, respectively. Moreover, derived from the total number of citations, the top 4 sources are “Construction and building materials”, “marine pollution bulletin”, “environmental pollution” and “science of total environmental”. Notably, this investigation would serve as a foundation for future scientometric studies on plastic sand. Furthermore, previous standard assessments were unable of producing scientific visualisation maps.

The article "A scientometric analysis approach on the plastic sand" was published in 2023. Journal: Heliyon.

**Table 1:** Publishing sites that released at least 15 publications on plastic sand from 2001 to June 2022.

S.No	Publication Source	Number of Publications	Number of Citations
1	Construction and building materials	134	3188
2	Marine pollution bulletin	63	1762
3	IOP conference series: materials science and engineering	56	98
4	Soil dynamics and earthquake engineering	53	519
5	IOP conference series: earth and environmental science	49	59
6	Science of the total environment	46	919
7	Geotechnical special publication	31	39
8	Environmental pollution	28	1213
9	Geotechnical and geological engineering	28	151
10	Materials	27	181
11	E3S web of conferences	27	37
12	Engineering structures	24	267
13	Soils and foundations	23	194
14	Materials today: proceedings	23	132

Fig. 6 shows the scientific visualisation of publishing sources that has at least 15 associated articles. The size of the frame box is related to the journal's influence on the document volume of the present study field; a larger box size specifies a greater influence. As an illustration, “Construction and building materials” frame box is much larger than the others frame box, indicating that it is a source of great significance in that subject. Three clusters were formed, each of which is characterized by a different color in the artwork (red, blue and green). The quantity of data contained in the research source or the number of times it is quoted in other publications that are similar [77] determines the formation of clusters. The VOSviewer classified journals according on co-citation trends of their articles published. For instance, the red cluster has 11 sources that have been mentioned numerous times in other publications that are essentially identical. Moreover, the links between closely spaced frames (journals) in a cluster are greater than those between widely spread frames. For example, “Construction and building materials” correlates more strongly with “Materials today: proceedings” than with “IOP conference series: materials science and engineering".

**Fig. 6:** Scientific visualisation of publishing sources that has at least 15 associated articles.

The article "A scientometric analysis approach on the plastic sand" was published in 2023. Journal: Heliyon.

### 3.3 Keywords

In analysis, one of the crucial parameters are the keywords as it determines and emphasise the fundamental subject of the study area [78]. “Co-occurrence” was selected as the “analysis type” for the evaluation, and “all keywords” was chosen as the “analysis unit”. The least number of times a keyword must be repeated in order for it to be maintained was set at 35, and only 130 of the original 15,033 keywords were kept. Table 2 presents a list of the top 20 words that appear most frequently in published literature on the topic. Sand, compressive strength, plastic, fibre reinforced plastic and reinforcement are the five keywords that come up the most frequently in the context of this area of research. Fig. 7 presents the visualisation map of keywords, illustrating their connections, co-occurrences, and density in a manner that is proportionate to the frequency with which they appear. The size of a keyword circle in Figure reflects how frequently it appears in articles, while the placement of the circle indicates how often it appears with other keywords. Additionally, the graph shows that the most important keywords have circles that are significantly larger than the others, which suggests that these keywords are very important to the study of plastic sand. The graph draws attention to word clusters in a way that demonstrates frequency with which they occurs together in a range of publications. The appearance of many keywords at the same time in previously published work serves as the basis for the color-coded grouping that is displayed. In the figure, there are three distinct colours that each indicate a different cluster: red, green, and blue. As may be seen in Fig. 8, various colours reflect various concentrations of keyword density. The density intensity of the colours red, green, and blue are listed from highest to lowest, with red indicating the maximum density intensity and blue being the lowest. Sand has more red markers, which indicates that it has a higher density concentration. Because of this revelation, prospective authors will have a better chance of selecting keywords that facilitate access to research on a certain subject.

**Table 2:** 20 of the most often used terms in plastic sand research.

S.No	Keyword	Occurrences
1	Sand	572
2	Compressive strength	254
3	Plastic	240
4	Fibre reinforced plastics	230
5	Reinforcement	217
6	Article	209
7	Soils	196
8	Plastics	186
9	Reinforced concrete	179
10	Reinforced plastics	174
11	Microplastic	168
12	Microplastics	167
13	Plastic waste	154
14	Particle size	142
15	Tensile strength	122
16	Polypropylenes	121
17	Concretes	120
18	Fibres	117
19	Water pollutant	112
20	Aggregates	111

The article "A scientometric analysis approach on the plastic sand" was published in 2023. Journal: Heliyon.

**Fig. 7:** Keyword analysis (scientific visualisation).

**Fig. 8:** Keyword analysis (density visualisation).

### 3.4 Authors

The impact in a given subject can be demonstrated by the number of citations received by a researcher [79]. For the assessment of authors, co-authorship was selected as the “kind of analysis” and “authors” were selected as the “unit of analysis”. The minimum number of papers per author was set at 10, and 36 of the 5719 authors satisfied this requirement. Table 3 displays the authors with the most published publications and citations in the study of plastic sand, as determined by data from the Scopus search engine. By dividing the overall number of citations by the total number of publications, the average number of citations for each author was calculated. When all parameters, including the publications count, and after that total citations in number, and the number of average citations, are counted in, it will be impossible to assess the effectiveness of a scientist. In contrast, the evaluation of the writer will be examined separately from each component, i.e. toal publications count, total citations count, and the average number of citations. Wang is the most prolific author with 30 works, followed by Wang, Zhang and Li with 27, 22 and 21 publications, respectively. In terms of total citations, Wu G. leads the field with 851, Wang with 821 and Zhao with 802 in the present study area. In addition, when the citations on average basis are compared, the following authors stand out: Zhao, Wu, Li and Dong has around 45, 43, 32 and 29 average number of citations. The association between writers with at least 36 publications and the most distinguished authors is depicted in Fig. 9. This investigation demonstrated number of authors that are linked by citations in the plastic sand research.

**Table 3:** Authors having a minimum of 10 publications in the field of RHA plastic sand by 2022.

S. No	Author	Total publications	Total citations	Average citations
1	Wang	30	821	27
2	Wang	27	143	5
3	Zhang	22	397	18
4	Li	21	153	7
5	Wang	21	158	8
6	Wu	20	851	43
7	Zhao	18	802	45
8	Dong	17	499	29
9	Zhang	17	141	8
10	Wang	16	156	10
11	Zhu	16	286	18
12	Benmokrane	15	202	13
13	Li	15	348	23
14	Li	14	442	32
15	Yang	14	339	24
16	Liu	13	180	14
17	Senetakis	13	134	10
18	Zhao	13	114	9
19	He	12	290	24
20	Li	12	105	9
21	Liu	12	148	12
22	Wu	12	68	6
23	Yang	12	121	10
24	Zhang	12	68	6
25	Zhang	12	46	4
26	Li	11	119	11
27	Wang	11	21	2
28	Wang	11	117	11
29	Chen	10	101	10
30	Li	10	68	7
31	Liu	10	120	12
32	Mohamed	10	146	15
33	Tong	10	279	28
34	Wang	10	40	4
35	Zhang	10	113	11
36	Zhang	10	92	9

**Fig. 9:** Visualisation of writers who have published publications in the relevant study field.

The article "A scientometric analysis approach on the plastic sand" was published in 2023. Journal: Heliyon.

### 3.5 Documents

The number of citations a publication receives often affects a particular study field. Papers that have been cited several times within their respective fields of research are regarded as pioneering work in those fields. The “type of analysis” was set to “bibliographic coupling” and “unit of analysis” was set to “documents” for the evaluation of documents. The minimum number of citations for a document was set at 80, and 38 out of 1895 papers met this threshold. The 5 most-cited works in the subject area of plastic sand, along with its authors and citation information, are included in Table 4. The work “Recycling of plastic solid waste: A state of art review and future applications” by Singh [80] earned 478 citations. Song, Talvitie and De Souza machado [[81], [82], [83]] acquired 438, 437 and 407 citations for their works, respectively, and were in the top 4. Until June 2022, however, just 9 works earned over 200 citations. Moreover, Fig. 10 depicts the map of related publications because of citations, along with the concentration of these papers in the present research topic. 38 of 21 publications were related by citations, as determined by the study. Fig. 10 depicts the mapping of associated articles based on citations. In addition, the density mapping (Fig. 11) demonstrates the increased density concentration of the top articles.

**Table 4:** Prior to June 2022, the top ten most-cited published plastic sand research publications.

S.No	Author	Name of Article	Total citations obtained
1	Singh [80]	Recycling of plastic solid waste: A state of art review and future applications	478
2	Song [81]	Combined Effects of UV Exposure Duration and Mechanical Abrasion on Microplastic Fragmentation by Polymer Type	438
3	Talvitie [82]	Solutions to microplastic pollution – Removal of microplastics from wastewater effluent with advanced wastewater treatment technologies	437
4	De Souza Machado [83]	Impacts of Microplastics on the Soil Biophysical Environment	407
5	Xiao [84]	Use of sea-sand and seawater in concrete construction: Current status and future opportunities	314
6	Shim [85]	Identification and quantification of microplastics using Nile Red staining	216
7	Wang [86]	Long-term durability of basalt- and glass-fibre reinforced polymer (BFRP/GFRP) bars in seawater and sea sand concrete environment	214
8	Coppock [87]	A small-scale, portable method for extracting microplastics from marine sediments	213
9	Li [88]	Effective uptake of submicrometre plastics by crop plants via a crack-entry mode	201
10	Michielssen [89]	Fate of microplastics and other small anthropogenic litter (SAL) in wastewater treatment plants depends on unit processes employed	172

The article "A scientometric analysis approach on the plastic sand" was published in 2023. Journal: Heliyon.

**Fig. 10:** Scientific mapping of published papers in the relevant subject field till June 2022 that are connected in terms of citations.

**Fig. 11:** Density visualisation of published papers in the relevant subject field till June 2022 that are connected in terms of citations.

### 3.6 Countries

The contribution of several regions/countries to plastic sand research is already substantial, yet there is room for improvement. The network map is created to facilitate access to plastic sand research regions for scientists. Countries were choosen as the “unit of analysis” and “bibliographic coupling” as the “kind of analysis”. The least number of documents per nation was set at 15, and 31 nations satisfied this threshold. The countries included in Table 5 have produced a minimum of 15 documents in the current topic of research. China, India, United States, Canada and Australia provided the most number of papers, 449, 217, 208, 97 and 90 respectively. Moreover, China, United States, India, Austraila and South Korea earned the most citations, with China obtaining 5672, United States receiving 3040, India receiving 2332, Australia obtaining 1997 and South Korea receiving 1391 citations, respectively. Fig. 12 presents a depiction of the scientific mapping as well as an illustration of the density of international connections made through citations. The size of a box in Fig. 12 corresponds to a country's influence on the topic research. The density visualisation map in Fig. 13 illustrates that the more engaging nations have a higher density. Emerging researchers will benefit from the statistical and graphical analysis of the participating nations since it will help them develop collaborations between scientists, form partnerships and exchange new methods and concepts. Scholars from different countries who are interested in furthering research on plastic sand have the opportunity to work together with experts in this area and take advantage from their extensive knowledge.

**Table 5:** Until June 2022, the leading nations based on published documents in the current study topic.

S. No	Name of Country	Total publications	Total citations received
1	China	471	5672
2	India	217	2332
3	United States	208	3040
4	Canada	97	958
5	Australia	90	1993
6	Iran	84	753
7	United Kingdom	82	1205
8	Germany	70	1282
9	Italy	58	1331
10	Japan	57	369
11	France	51	613
12	Brazil	50	389
13	Indonesia	49	220
14	South Korea	48	1391
15	Malaysia	45	424
16	Turkey	45	318
17	Poland	45	167
18	Algeria	41	360
19	Spain	40	328
20	Netherlands	32	644
21	Iraq	32	378
22	Russian Federation	32	334
23	Nigeria	27	148
24	Egypt	26	244
25	Viet Nam	24	311
26	Saudi Arabia	23	190
27	Portugal	18	141
28	Greece	17	265
29	Pakistan	17	186
30	South Africa	16	115
31	Mexico	16	60

The article "A scientometric analysis approach on the plastic sand" was published in 2023. Journal: Heliyon.

**Fig. 12:** Network visualisation of nations having a minimum of 15 publications in the relevant study field until June 2022.

**Fig. 13:** Density visualisation of nations having a minimum of 15 publications in the relevant study field until June 2022.

Moreover, previous researchers has also suggested that between 2011 and 2013, China nation has utilised more sand for the production of concrete than the United States utilised throughout the entirety of the 20th century [21]. Two-thirds of the $94,000 billion anticipated to be invested on infrastructure worldwide from 2015 to 2030 will be spent in developing nations such as China and India [15], with modern fast industrialization and urbanization being the primary drivers of this expansion in the Asia-Pacific region. It is anticipated that the need for sand will continue to rise; specifically, it is anticipated that India's demand for sand would triple during the next several decades if it maintains the same growth track as China [90].

## 4 Discussion and future perspective

This paper provides a statistical and cartographic summary of the current literature on plastic sand. The standard review study that is done manually has restricted comprehensiveness and a less precise interrelationship between distinct portions of the literature. In addition, this study evaluates the journals with the most published papers, the most frequently used keywords in published studies, the primary contributing nations, and the articles and authors with the most citations in the plastic sand research field. The analysis of plastic sand by countries identified that most of the studies have been conducted in China, India and United State. The difficulties they confront with waste management might be one of the reasons why academics in these fields are so interested in plastic sand. The UNEP observed in 2021 [91] that waste collection facilities in the majority of African nations are inadequate. For instance, the average percentage of municipal solid waste (MSW) collection is around 55%, while 13% of MSW was found in Africa is plastic garbage. Even though 70–80% of MSW is recyclable, only 4% of the MSW is found to be recycled in Africa [91]. Instead of being motivated by public or private sector activities, Africans have started recycling more because of the continent's socioeconomic necessities brought on by widespread poverty and unemployment. Problems with waste management can be resolved by adding plastic waste and sand in the construction sector. Furthermore, the literature and their linkage, which were based on the number of citations, revealed the countries that were most engaged and contributed the most in terms of publications. Young researchers will find it easier to create scientific partnerships, develop joint projects, and share new approaches and ideas with the help of the data, which uses statistical and graphical depictions of the countries that contributed to the project. Researchers from countries that are interested in advancing the study of plastic sand can collaborate with specialists in the subject in order to benefit from their knowledge and experience.

The article "A scientometric analysis approach on the plastic sand" was published in 2023. Journal: Heliyon.

In order for plastic sand bricks to be commercially viable as an alternative building material, its production and utilisation must be cost-effective. Moreover, according to one study, the use of PET waste in construction materials decreases the cost of such products [92]. Despite the fact that waste plastic is quite inexpensive, this does not indicate that plastic sand will replace traditional building materials any time soon. In some countries, the process of collecting, transporting, and storing waste plastic might be considered impractical. Therefore, economic assessment studies must be conducted to analyse the viability in construction sector for adopting plastic sand [92]. In addition, studies on the industrialization of the use of plastic sand are required. As without such investigations, the use of plastic sand in the construction sector would only exist in theory as viable alternatives to conventional building materials. The relevance of evaluating the economic viability of plastic sand that has been utilised in bricks and also in blocks is supported by the fact that these blocks and bricks manufactured in the concrete sector was valued at 1700.55 billion (USD) in 2019 and is expected to reach 2563 billion (USD) by 2027 [93]. Therefore, there is need to study on the properties of the different types of plastic waste and sand available around the globe. So that they can be utilised by industries which will help in environment sustainability. There has not been any study done in the past that has investigated whether or not plastic sand are flammable or whether or not they are resistant to fire, both of which are essential characteristics for the use of plastic sand in the industry. The only people to assert that waste plastic sand bricks are easily flammable were Selvamani et al. [94]. But the true findings of their results were not revealed. Moreover, Abdel Tawab et al. [95] conducted study on the thermal conductivity of the bricks that were made from plastic sand. They discovered that the bricks thermal conductivity declined as the plastic amount that is contained within the bricks rises. Therefore, more in depth knowledge is required to be covered in this field of research.

The article "A scientometric analysis approach on the plastic sand" was published in 2023. Journal: Heliyon.

Plastics and sand are extremely valuable materials that offer countless benefits to individuals and society. Due of the limited biodegradability of plastics, this problem will remain for millennia [96]. This article describes current advancements in the utilisation of plastic and sand mixes. Numerous civil engineering uses for plastic sand bricks include precast bricks, partition walls, roof tiles, canal linings, and paving bricks. Notable about these applications is that they help in the disposal of non-biodegradable plastic wastes that collect across the world. Thus, the purpose of the study is to highlight the necessity for more research and development of plastic sand. Plastic sand building materials (e.g., bricks, blocks, tiles) will produce a sustainable alternative material, reduce prices, enhance performance, and encourage sustainable waste management in the construction sector.

## 5 Conclusion

Plastics and sand are both incredibly important commodities that provide a myriad of advantages to both people and society as a whole. This problem will not be solved for millennia since plastics have a limited capacity for biodegradation. This article discusses recent developments in the use of plastic and sand mixtures. The purpose of this research was to conduct a scientometric analysis of the existing literature on the topic of plastic sand in order to assess a variety of characteristics. The Scopus search engine database was used for 4512 pertinent articles, and the findings were evaluated with the VOSviewer application. This investigation produced the following outcomes:

• An examination of published sources comprising documentation on plastic sand revealed the leading five sources to be “Construction and building materials”, “marine pollution bulletin”, IOP conference series: materials science and engineering”, “soil dynamics and earthquake engineering” and “IOP conference series: earth and environmental science” contain 134, 63, 56, 53 and 49 papers, respectively. Moreover, based on the total number of citations, the top four sources are “Construction and building materials”, “marine pollution bulletin”, “environmental pollution” and “science of total environmental” having citations 3188, 1762, 1213 and 919, respectively.
• A keyword analysis of the topic of research reveals the five most often occurring terms are sand, compressive strength, plastic, fiber reinforced plastics and reinforcement. The occurrence of the top 5 keywords in the published paper were as follows; 572 (sand), 254 (compressive strength), 240 (plastic), 230 (fiber reinforced plastics) and 217 (reinforcement).
• After doing author analysis, the researchers found that only 36 authors had contributed to at least 10 different plastic sand research articles. The best writers were ranked based on how many publications they have put out, how many citations they have received, and how many citations they receive on average. Wang Z. is the most prolific author with 30 works, followed by Wang, Zhang and Li with 27, 22 and 21 publications, respectively. In terms of total citations, Wu G. leads the field with 851, Wang with 821 and Zhao with 802 in the present study area. In addition, when average citations are compared, the following authors stand out: Zhao, Wu, Li and Dong has around 45, 43, 32 and 29 average citations.
• According to a review of articles containing information about plastic sand; “Recycling of plastic solid waste: A state of art review and future applications” by Singh earned 478 citations. Song, Talvitie and De Souza machado acquired 438, 437 and 407 citations for their works, respectively, and were in the top 4. From 2001 until June 2022, however, just 9 works earned over 200 citations.
• On the basis of the main nations involvement in plastic sand research, it was concluded that only 32 countries published atleast 15 papers. China, India, United States, Canada and Australia provided the most number of papers, 449, 217,208, 97 and 90 respectively. Moreover, China, United States, India, Australia and South Korea earned the most citations, with China obtaining 5672, United States receiving 3040, India receiving 2332, Australia obtaining 1997 and South Korea receiving 1391 citations, respectively.
• Based on the review from 2001 to June 2022, it was apparent that the construction industry has been the most prevalent user of plastic sand, seeing the top 5 keywords and documents citations.
• Usage of plastic sand in the construction industry would also contribute to green construction and environmental sustainability.
• The vast majority of potential uses for plastic sand have not yet been fully explored, and further research is necessary before expanding the scope of their applicability.

The article "A scientometric analysis approach on the plastic sand" was published in 2023. Journal: Heliyon.

## 6 Limitations and future recommendations

Due to its data-driven methodology, this study will be influenced by the quality of the data collected. Even if the data were acquired using a scientometric data retrieval method, the logical combination of phrases cannot guarantee that alternative articles were also collected, since some studies may use the term “discarded material” rather than “waste material”. In addition, the Scopus database was utilised because it had more papers than the Web of Science database. When non-English articles are considered, the frequency of search phrases may increase. In addition, VOSviewer grouped and displayed the keywords according to their co-occurrences in the mined articles. The contents of the clusters corresponded closely to the topics of the clusters to which they belonged. When comparable terms are stored in separate clusters, the data's sensitivity is shown. However, given the study's limitations, it is doubtful that the findings and conclusions would undergo much modification. Future research should be undertaken on a regular basis to examine the limitations of utilising data from several sources, search methods, and indications.

## Author contribution statement

All authors listed have significantly contributed to the development and the writing of this article.

## Funding statement

This work was supported by the 10.13039/501100002385Ministry of Higher Education of Malaysia and 10.13039/501100005417Universiti Teknologi Malaysia [5F545,5F365, 4J224, 4B499].

## Data availability statement

Data included in article/supp. material/referenced in article.

## Declaration of interest's statement

The authors declare no conflict of interest.
